This article has been retracted.

# Medication Non-Adherence among Patients with Heart Failure

**DOI:** 10.7759/cureus.5346

**Published:** 2019-08-08

**Authors:** Zahid U Rehman, Arsalan K Siddiqui, Musa Karim, Haris Majeed, Muhammad Hashim

**Affiliations:** 1 Miscellaneous, National Institute of Cardiovascular Diseases, Karachi, PAK; 2 Miscellaneous, Aga Khan University Medical College, Aga Khan University Hospital, Karachi, PAK; 3 Cardiology, National Institute of Cardiovascular Diseases, Karachi, PAK

**Keywords:** morisky medication adherence scale, heart failure, medication, adherence

## Abstract

Introduction

Poor adherence or non-adherence to the prescribed medications among heart failure (HF) patients is a common problem. This leads to hospital admission due to increased HF exacerbations, reduced physical function, and even death. The study was conducted to assess the heart failure medication adherence level, using Morisky Medication Adherence Scale (MMAS-8), among heart failure patients visiting the adult cardiology department of a tertiary care cardiac center in Karachi.

Methods

This cross-sectional study included patients diagnosed with heart failure visiting for the follow-up to both inpatient and outpatient departments of a tertiary care cardiac center of Karachi, Pakistan. Medication adherence level was assessed using a validated Morisky Medication Adherence Scale (MMAS-8). The total MMAS-8 score was calculated by adding all of the 8 individual question scores and patients with a score of eight were classified as adherent, otherwise non-adherent.

Results

A total of 200 patients were included in this study, out of which 61.5% (123) were male and 38.5% (77) were female. More than half, 54% (108), of the patients were rural residents and majority were Urdu (39.5%) speaking followed by Sindhi (19.5%) and Pashto (19.0%) speaking. Almost all, 99.5% (199) were married and 52% (104) patients were uneducated. Overall 76.5% (153) were adherent to the prescribed medication. And reaming 23.5% (47) were moderately adherent with MMAS-8 score of seven and six. Non-adherence to the prescribed medication is more common among rural residents and uneducated patients.

Conclusion

Non-adherence to the prescribed medication was observed in a significant number of heart failure patients (23.5%) in our population, and it was more common observation for the patients with rural residence and uneducated. It is important to counsel the patients about the importance of medication adherence to marginalize the re-hospitalization and complications these patients.

## Introduction

Heart failure (HF), a chronic cardiac disease characterized by high mortality and hospitalization, carries a significant burden of disease throughout the world, especially in Pakistan [1-2]. A state in which the heart fails to pump blood into systemic circulation sufficiently, many risk factors such as smoking, hypertension, alcoholism, and previous history of cardiac disease have been delineated [1]. In Pakistan, a high percentage of coronary heart disease leads to HF, and this is attributed to the lack of treatment and/or lack of medicine compliance [3]. Medical management and adherence in the form of lipid-lowering, anti-thrombotic therapy, and mitigation of risk factors have constantly been shown to predict the rate of hospitalization [4]. Similarly, the American College of Cardiology, the American Heart Association and the European Society of Cardiology guidelines implore medication adherence due to its reductive potential in regards to morbidity and mortality in HF [5-6].

Though increasingly complex, medical management and mitigation of risk factors based on the 2016 American College of Cardiology Foundation / American Heart Association Guideline recommendations are fundamental in HF patients with decreased ejection fraction (EF) [7]. Such treatment, including first-line anti-arrhythmias and beta-blockers, has shown to decrease the occurrence of shocks or other emergencies, thus significantly decreasing the rates of re-hospitalization [8-9].

In known HF patients, advancement in life quality as well as life-span are paramount and are significantly dependent on treatment. Unfortunately, however, medical adherence to medication remains less than what desired and required. Studies have demonstrated that close to 25% of patients with HF do not consistently take the relevant prescribed medications [10-11]. Moreover, it has also been shown that roughly half of the patients with chronic HF do not take the clinically effective dosages of medication, in regards to frequency [1]. In this study, we hope to delineate the factors leading to decreased medical adherence in HF patients, whether that be a gap in patient understanding, symptomatic changes in patients, or availability of medications. The purpose of this study was to assess HF medication adherence level among the patients visiting the outpatient department of a tertiary care cardiac center.

## Materials and methods

This cross-sectional study included patients of either gender, between 40 to 80 years of age, and diagnosed with HF, visiting for follow-up in both inpatient and outpatient departments of a tertiary care cardiac center at Karachi, Pakistan. Patients with congenital heart disease or valvular heart diseases were excluded from the study. Prior to inclusion in the study, verbal informed consent was taken from all the patients. Demographic variables such as gender, age (years), residence (urban/rural), mother tongue, marital status, highest education, and the time since HF were recorded. Medication adherence level was assessed using a validated Morisky Medication Adherence Scale (MMAS-8) [12]. The tool consists of eight questions, and scoring was done according to an already developed method, in which the total score is eight. For questions one through seven, there was a score of zero for every “yes” response and one for every “no” response, while the eighth question was assessed on five-point scale from “never/rarely’ to “all the time”, a score of one was assigned to “never/rarely’ response and zero for all other responses. MASS-8 scale is presented in Figure 1.

**Figure 1:** Morisky Medication Adherence Scale (MMAS-8) [12]

The total MMAS-8 score was calculated by adding all of the eight individual question scores and patients with a score of eight were classified as adherent, otherwise non-adherent. Data were entered and analyzed using IBM SPSS Statistics for Windows, Version 21.0. (IBM Corp., Armonk, NY, US). Continuous variables were expressed as mean ± standard deviations or median (inter-quartile range), and categorical variables were expressed as frequency and percentages. The chi-square test was applied to assess the association of medication adherence with various demographic variables. Multivariate logistic regression analysis was performed to identify the predictors for the non-adherence to the HF medication. Clinically significant variables such as gender, age, duration since diagnosis, education of the patient, and rural residence were taken as explanatory variables for the multivariate logistic regression analysis. *P*-values ≤ 0.05 was considered as statistically significant.

## Results

A total of 200 patients were included in this study, out of which 61.5% (123) were males and 38.5% (77) were females. The mean age of the patient was 56.86 ± 12.74 years ranging over 20 to 85 years with the majority of the patients, 68.5% (137), above 50 years of age. More than half, 54% (108), of the patients were rural residents and majority were Urdu (39.5%) speaking followed by Sindhi (19.5%) and Pushto (19.0%) speaking. Almost all, 99.5% (199) were married and 52% (104) patients were uneducated. The mean duration since the diagnosis of HF was 51.85 ± 26.83 months, ranging over one to 192 months.

Overall, 76.5% (153) were adherent to the prescribed medication. The remaining 47 were moderately adherent with an MMAS-8 score of seven in 46 patients and six in one patient. Medication adherence by baseline demographic characteristics is presented in Table 1. Non-adherence to the prescribed medication was more common among rural residents and uneducated patients.

**Table 1:** Medication adherence by baseline demographic characteristics *significant at 5%

Characteristics	Medication Adherence		
	Adherent	Non-adherent	p-value
Gender			
Male	58 (37.9%)	19 (40.4%)	0.756
Female	95 (62.1%)	28 (59.6%)	
Age			
Up to 40 years	17 (11.1%)	5 (10.6%)	0.025*
41 to 60 years	76 (49.7%)	23 (48.9%)	
More than 60 years	60 (39.2%)	19 (40.4%)	
Residency			
Rural	75 (49%)	33 (70.2%)	0.011*
Urban	78 (51%)	14 (29.8%)	
Mother tongue			
Urdu	60 (39.2%)	19 (40.4%)	0.882
Sindhi	31 (20.3%)	7 (14.9%)	0.412
Pushto	32 (20.9%)	7 (14.9%)	0.362
Hindko	11 (7.2%)	5 (10.6%)	0.446
Punjabi	8 (5.2%)	6 (12.8%)	0.077
Balochi	7 (4.6%)	2 (4.3%)	0.926
Others	4 (2.6%)	1 (2.1%)	0.852
Education			
Graduate	2 (1.3%)	1 (2.1%)	0.686
Intermediate	9 (5.9%)	1 (2.1%)	0.302
Matric	35 (22.9%)	8 (17%)	0.393
Middle	31 (20.3%)	4 (8.5%)	0.064
Primary	4 (2.6%)	1 (2.1%)	0.852
Uneducated	72 (47.1%)	32 (68.1%)	0.012*
Time Since heart failure			
Upton 48 months	88 (57.5%)	26 (55.3%)	0.790
More than 48 months	65 (42.5%)	21 (44.7%)	

Multivariate logistic regression analysis for non-adherence to the medication of heart failure are presented in Table 2. The rural residence was found to be an independent predictor of medication non-adherence with an adjusted odds ratio (OR) of 2.19 [1.04 - 4.61].

**Table 2:** Predictors of non-adherence to the medication of heart failure *significant at 5%

Predictors	Odds Ratio (OR)	95% Confidence Interval	P-value
Male	1.03	0.51 to 2.07	0.941
Age ≥60 years	1.20	0.6 to 2.42	0.606
Rural residents	2.19	1.04 to 4.61	0.039*
Uneducated	1.92	0.92 to 4	0.081
≥48 months since diagnosis	0.78	0.39 to 1.55	0.477
Constant	0.13	-	<0.001*

## Discussion

Rehospitalization due to medication non-adherence remains the leading problem in heart failure patients across the globe. This study was conducted to determine the level of adherence to the prescribed medication among patients with HF. We observed that a significant number of patients (23.5%) were non-adherent to the prescribed medication for HF. Despite its utmost importance, there is a paucity of reliable local data on medication adherence among the HF patients in our population. Such studies will help healthcare professionals to design targeted interventions and patient counseling strategies to restrain this public health issue in our population.

In Pakistan, especially in the urban areas, there are several HF patients who are living compromised life and rehospitalized whenever symptoms get worse due to non-adherence to the heart failure medications. Six out of 10 patients reported sometimes forgetting to take medication according to Morisky Medication scale [8]. An observational survey study published in December 2010 in the same population reported that out of 267 patients, 73 (27.3%) were compliant while 194 (72.7%) were noncompliant. They identified the main reasons for non-compliance are financial, social, and medical issues [13].

Proper counseling and targeted interventions to increase the medication adherence level are needed as medication non-adherence leads to increased rates of mortality, morbidity, and hospital readmissions [14]. Various predictors of medication adherence were also identified such as patient’s age, gender, ethnicity, disease characteristics, type of disease, number of medicines, and frequency of visits to health-care professionals, satisfaction with treatment and forgetfulness, which can reduce medication adherence [15]. In our study, non-adherence to the prescribed medication was more common among rural residents and uneducated patients. Non-adherence to the prescribed medications is not only limited to the heart failure patients, but some studies on medication non-adherence conducted in Pakistan also estimated the high percentage of poor medication adherence among patients with various other medical conditions or diseases such as hypertension, or myocardial infarction, etc. [15-18].

## Conclusions

Non-adherence to the prescribed medication was observed in a significant number of HF patients (23.5%) in our population, and it was more common observation for the patients with rural residence and uneducated. Association of medication non-adherence and frequent re-hospitalization and other complications among heart failure patients is evident in the literature. It is important to counsel the patients about the importance of medication adherence to marginalize the re-hospitalization and complications in these patients.
